This article has been retracted.

# Expression of Tspan8 in Patients with Intrahepatic Cholangiocarcinoma and Its Relationship with Clinicopathological Features and Prognosis

**DOI:** 10.1155/2021/7475938

**Published:** 2021-10-21

**Authors:** Zhenhua Tan, Renrui Wan, Minzhi Chen, Ping Xie, Peng Li, Yan Shen, Zhiping Pan, Hai Qian

**Affiliations:** ^1^Department of Hepatopancreatobiliary Surgery, Huzhou Central Hospital, Affiliated Central Hospital Huzhou University, Huzhou, Zhejiang 313000, China; ^2^Graduate School of Zhejiang University, Hangzhou, Zhejiang 310000, China; ^3^Department of Operating Room, Huzhou Central Hospital, Affiliated Central Hospital Huzhou University, Huzhou, Zhejiang 313000, China; ^4^Department of General Surgery, Huzhou Central Hospital, Affiliated Central Hospital Huzhou University, Huzhou, Zhejiang 313000, China

## Abstract

The incidence and mortality of intrahepatic cholangiocarcinoma (ICC) are increasing worldwide. High invasion and metastasis are one of the main causes of death in patients. The selection of reasonable and effective molecular markers to evaluate the prognosis of patients with ICC has important clinical guiding significance. In this study, the expression of Tspan protein in ICC and normal tissues was compared, the correlation between Tspan expression and pathological features of patients was analyzed by the logistic regression model using multivariate analysis, and the relationship between Tspan8 expression and prognosis of ICC patients was analyzed by the Kaplan–Meier survival curve. The results showed that Tspan8 is highly positive in ICC tissues, TNM stage, degree of tumor differentiation, lymph node metastasis, and Tspan8 protein expression were independently correlated, and the overexpression of Tspan was associated with the prognosis of ICC invasion and metastasis. This provides a new idea for clinical treatment.

## 1. Introduction

Intrahepatic cholangiocarcinoma (ICC) is adenocarcinoma originating from secondary bile ducts and their branched epithelium, accounting for about 10% of primary liver cancers [1]. Bile duct stones, cirrhosis, and HBV infection are important factors for ICC. Studies have shown that the 5-year survival rate of ICC patients is about 5%–10%, and the prognosis of most patients is poor [2]. However, at present, the prediction of ICC disease stage and prognosis is mainly based on the pathological characteristics of tumors, there is a lack of information at the molecular level, and the research on adjuvant therapy such as targeted drugs cannot provide more information [3]. Therefore, it is of great significance to find and identify effective biomarkers, explore their mechanisms in the occurrence and development of ICC, and provide effective molecular targets for the early diagnosis, treatment, and prognosis assessment of ICC.

Tspan8 is a conserved small molecule membrane protein encoded by TSPAN8 gene, which is composed of 237 amino acid residues [4]. This protein is a member of the transmembrane 4 superfamily/tetraspanin (TM4SF/Tspan) [5]. Tspan8 plays multiple roles in human body. It can not only participate in the regulation of multiple biological functions such as tumor metastasis, viral infection, platelet aggregation, and immune response but also affect a variety of biological behaviors including the adhesion, migration, differentiation, and malignant transformation of cells [6]. Previous studies have confirmed that Tspan8 is highly expressed in various solid tumors such as liver cancer, esophageal cancer, and melanoma and has significant effects on promoting tumor invasion and metastasis. However, there are few studies on its role in ICC and the correlation between its clinical changes and the prognosis of ICC patients is not clear [7]. Therefore, the focus of this study is to observe the expression changes of Tspan8 in patients with intrahepatic cholangiocarcinoma and its relationship with clinicopathological features and prognosis, aiming to provide a corresponding theoretical basis for clinical application research, which is reported as follows.

## 2. Materials and Methods

### 2.1. General Data

A total of 100 ICC patients admitted to our hospital from January 2015 to December 2018 were included as the research objects. Among them, there were 56 males and 44 females, with the average age of 45.67 ± 2.31 years. There were 41 cases in stage I + II and 59 cases in stage III + IV of TNM stage. The average tumor diameter was 5.24 ± 2.17 cm. Preoperative carcinoembryonic antigen (CEA) was ≥5 ng/mL in 67 cases and <5 ng/mL in 33 cases. Also, there were 38 cases of lymph node metastasis and 40 cases of vascular tumor thrombus.

All study subjects underwent radical surgical resection, and tumor tissues of intrahepatic cholangiocarcinoma and adjacent normal bile duct tissues more than 5 cm away from the tumor were taken to serve as the ICC group and the normal tissue group, respectively.

### 2.2. Inclusion Criteria

The inclusion criteria were as follows: (i) ICC is confirmed by pathological examination, (ii) patients without history of radiotherapy or chemotherapy before enrollment, (iii) patients with complete case and follow-up data, and (iv) patients without cardiac or cerebrovascular diseases.

### 2.3. Exclusion Criteria

The exclusion criteria were as follows: (i) patients whose perioperative death or nontumor-related death occurred during follow-up, (ii) patients with mixed liver cancer, (iii) patients with previous history of biliary surgery, and (iv) patients with cognitive and mental disorders.

### 2.4. Tspan8 Detection Method

All the collected tissues were embedded in paraffin, and the expression level of Tspan8 protein was detected by immunohistochemistry (IHC) after 4 *μ*m continuous sections were made. Tspan8 antibody was purchased from Abcam, China, with a dilution of 1 : 500. According to the instructions of immunohistochemistry kit and DAB reagent kit, PBS buffer was used to replace primary antibody as negative control. First, paraffin sections were routinely dewaxed, cleaned, and sealed. After completion, diluted Tspan8 primary antibody was dropped and incubated overnight at 4°C. On the second day, wash the tissue in PBS 3 times, 5 min each time, dry the tissue around PBS, and then drop secondary antibody. The samples were washed in PBS 3 times, 5 min each time. The PBS around the tissues was dried, and a color developing agent was added. DAB kit, hematoxylin, and blue-back solution were used for staining. Finally, the slices were dehydrated with gradient ethanol, transparent with xylene, and sealed with neutral resin.

There were positive and negative controls in each group of experiments, each section was viewed randomly, and tspan8 expression was judged comprehensively based on the percentage of positive cells to the total population of the same cells and the intensity of the staining. For high expression, the average number of positive staining cancer cells in tumor level sections was ≥50%; for low expression, the average number of positive staining cancer cells was <50% [8].

### 2.5. Data Collection

The medical records of all patients were collected, and the gender, age, TNM stage, tumor diameter, preoperative CEA, vascular tumor thrombus, lymph node metastasis, preoperative CA199, smoking history, drinking history, and degree of tumor differentiation were statistically analyzed. All subjects were continuously followed up for 3 years. The follow-up period was until April 30, 2021, and the follow-up mode was dominated by hospital review. Follow-up intervals were as follows: every 2 months in the first year, every 3 months in the second year, and every 6 months in the third year.

### 2.6. Statistical Methods

All data were processed with SPSS 22.0 statistical software, and GraphPad Prism 8 was used to make statistical graphs. Measurement data are expressed as mean ± standard deviation (±*s*), and the independent sample *t*-test is used for comparison between groups. Count data are expressed as (*n* (%)), and the chi-square (*χ*^2^) test is performed. The Kaplan–Meier survival curve was used to analyze the relationship between Tspan8 expression and prognosis in ICC patients, and the log-rank test was used for comparison. Multivariate logistic regression analysis was used to study the risk factors of coronary artery disease in young patients with AMI. The difference is statistically significant when *P* < 0.05.

## 3. Results

### 3.1. Comparison of Tspan8 Expression in ICC and Paracancer Normal Tissues

In the ICC group, 61 cases were positive and 39 cases were negative, with a positive rate of 61.00%. In the normal tissue group, 32 cases were positive and 68 cases were negative and the positive rate was 32.00%. The positive rate of Tspan8 in the ICC group was higher than that in normal tissue group, and the difference was statistically significant (*χ*^2^ = 16.903, *P* ≤ 0.001; Figure 1).

The positive expression of Tspan8 protein was mainly found in the cell membrane and some cytoplasm of tumor cells. Tspan8 protein was brownish yellow or dark brown in ICC samples, and the number of positive cells was significantly greater than 50%. However, the staining intensity and positive cell number of Tspan8 protein were significantly decreased or no positive expression was observed in the paired adjacent nontumor tissues (Figures 2(a) and 2(b)).

### 3.2. Relationship between Tspan8 Protein Expression and Clinicopathological Features of ICC Patients

The positive expression rate of Tspan8 protein in patients with preoperative CEA ≥ 5 ng/mL was higher than that in patients with preoperative CEA < 5 ng/mL. The positive expression rate of Tspan8 protein in patients with low tumor differentiation was higher than that in patients with medium and high tumor differentiation. The positive expression rate of Tspan8 protein in patients with lymph node metastasis was higher than that in patients without lymph node metastasis. The positive expression rate of Tspan8 protein in TNM stage III + IV was higher than that in TNM stage I + II. The comparison was statistically significant (*P* < 0.05).

However, there was no correlation between Tspan8 expression and gender, age, tumor diameter, preoperative CEA, vascular tumor thrombus, preoperative CA199, smoking history, and drinking history of ICC patients (*P* > 0.05; Table 1).

### 3.3. Logistic Regression Analysis of Tspan8 Protein Expression and Clinical Clinicopathological Features of ICC Patients

Logistic regression analysis showed that TNM stage, degree of tumor differentiation, lymph node metastasis, and Tspan8 protein expression were independently correlated (*P* < 0.05; Table 2).

### 3.4. Analysis of the Relationship between Tspan8 Protein Expression and Prognosis of ICC Patients

As of April 30, 2021, 46 of the 100 ICC patients died and 5 were lost to follow-up, with an overall mortality rate of 48.42%. The median survival time of patients with positive Tspan8 expression was 24.0 months and that of patients with negative Tspan8 expression was 31.0 months, with log-rank test *P*=0.002, and the difference was statistically significant (*P* < 0.05; Figure 3).

## 4. Discussion

ICC is the second most common primary malignant tumor in the liver [9]. Its occurrence and metastasis are multifactorial and multistep complex, with sequential processes involving changes at multiple levels including genes, signaling pathways, and epigenetics. TM4SF/Tspan is a special cell membrane glycoprotein, which widely exists in mammalian body. Invasion and migration are the important biological characteristics of malignant tumors [10, 11]. In recent years, studies have found that some members of TM4SF family can affect the invasion and migration of tumors, so these molecules have gradually become candidates for therapeutic targets.

Tspan8 is composed of transmembrane proteins, and many previous studies have revealed the mechanism of Tspan8 in various tumor diseases [12]. For example, Tspan8 can promote the metastasis and progression of esophageal cancer by upregulating the expression of ADAM12 [13]. It can influence environmental signals to promote the growth and invasion of colon cancer cells [14]. It can also inhibit apoptosis, induce cell cycle arrest of NSCLC, and accelerate tumor development [15]. This study compared the expression of Tspan protein between ICC and normal tissues, and the correlation between Tspan8 protein expression and pathological features of patients was analyzed. The results showed that Tspan was highly expressed in ICC tissue, and the TNM stage, degree of tumor differentiation, lymph node metastasis, and Tspan8 protein expression were independently correlated (*P* < 0.05), suggesting that Tspan8 expression was closely related to the occurrence and development of ICC. The higher the expression level of Tspan8 in ICC tissues, the higher the TNM stage and malignant differentiation degree of patients. Also, combined with previous data, we thought that Tspan affects ICC tumor cell growth and lymphatic metastasis mainly by integrins, MMPs, and transmembrane domain (TM).

Integrin is an important associated molecule of Tspan8 [16]. The combination of integrin and Tspan8 can act on multiple downstream targets such as ERK, AKT, and JNK, induce tumor angiogenesis by activating the vascular endothelial growth factor signaling pathway, and promote tumor cells to penetrate the vascular endothelial barrier, thereby accelerating tumor cells to metastasize to distant regions [17–19]. Meanwhile, Tspan8 can promote MMPs to secrete epidermal growth factor (EGF), transforming growth factor-*β* (TGF-*β*), insulin-like growth factor (IGF), and other growth factors and play a multifaceted role [20]. On the one hand, it accelerates the division of tumor cells; on the other hand, it degrades the extracellular matrix and promotes the spread of cancer cells beyond the extracellular matrix barrier [21]. In addition, there are studies showing that Tspan8 controls the proliferation and migration of tumor cells by fixing TM on the cell membrane. Moreover, TM can combine different molecules including integrins, cell surface receptors, and metalloproteases to form a quadruple protein network [22–24].

Zhang et al. [25] suggested that Tspan8 could be used as a promising biomarker for diagnosis and prognosis of colorectal cancer. Similarly, Tang et al. [26] found that the high expression of Tspan8 was associated with poor overall survival in 150 patients with renal clear cell carcinoma in the Kaplan–Meier analysis and log-rank test in a clinical follow-up study, thus suggesting a potential role of Tspan8 in prognosis and targeted therapy. In this study, Kaplan–Meier survival curve analysis showed that Tspan8 overexpression was closely related to the survival time of ICC patients, and the overall survival rate of ICC patients with high positive Tspan8 expression was lower, which suggested that clinical monitoring of Tspan expression may help predict the clinical prognosis of patients. This provides strong data for early biotherapy. Based on this, we believe that it is significant to routinely evaluate Tspan8 immunohistochemical staining in patients with ICC after surgery, which can provide strong support for reducing postoperative recurrence rate and mortality rate of patients.

In conclusion, Tspan8 is highly positive in ICC tissues and overexpression of Tspan was associated with the clinicopathological features and prognosis of ICC invasion and metastasis. Also, Tspan8 could be used as a therapeutic target for predicting the prognosis of ICC patients.

## Figures and Tables

**Figure 1:** Expression of Tspan8 in cancer tissues and adjacent normal tissues of patients with ICC.

**Figure 2:** Immunohistochemical staining showed Tspan8 protein expression in an (a) ICC tissue and (b) paired paracancer normal tissue.

**Figure 3:** Survival curves of patients with positive and negative Tspan8 expression.

**Table 1:** Relationship between Tspan8 protein expression and clinicopathological features of ICC patients (*n*, $\bar{x}$ ± *s*).

Clinicopathological features	Total number of cases (*n* = 100)	Tspan8 protein			
		Negative	Positive	*χ* ^2^	*P*
*Age*					
≥60 years old	54	22 (56.41)	32 (52.46)	0.150	0.699
<60 years old	46	17 (43.59)	29 (47.54)		

*Gender*					
Male	56	21 (53.85)	35 (57.38)	0.120	0.729
Female	44	18 (46.15)	26 (42.62)		

*Preoperative CEA*					
≥5 ng/mL	67	16 (41.03)	51 (83.61)	19.509	≤0.001
<5 ng/mL	33	23 (58.97)	10 (16.39)		

*Preoperative CA199*					
≥34 U/mL	69	26 (66.67)	43 (70.49)	0.163	0.687
<34 U/mL	31	13 (33.33)	18 (29.51)		

*Tumor diameter*					
<4 cm	45	16 (41.03)	29 (47.54)	0.408	0.523
≥4 cm	55	23 (58.97)	32 (52.46)		

*Degree of tumor differentiation*					
Low differentiation	40	9 (23.08)	31 (50.82)	7.629	0.006
Moderate and high differentiation	60	30 (76.92)	30 (49.18)		

*Lymph node metastasis*					
Yes	38	11 (28.21)	27 (44.26)	2.603	0.107
No	62	28 (71.79)	34 (55.74)		

*TNM stage*					
I + II stage	41	27 (69.23)	14 (22.95)	21.064	≤0.001
III + IV stage	59	12 (30.77)	47 (77.05)		

*Vascular tumor thrombus*					
Yes	40	18 (46.15)	22 (36.07)	1.009	0.315
No	60	21 (53.85)	39 (63.93)		

*Smoking history*					
Yes	58	20 (51.28)	38 (62.30)	1.184	0.276
No	42	19 (48.72)	23 (37.70)		

*Drinking history*					
Yes	46	16 (41.03)	30 (49.18)	0.637	0.425
No	54	23 (58.97)	31 (50.82)		

**Table 2:** Logistic regression analysis of Tspan8 protein expression and clinical clinicopathological features of ICC patients.

Influencing factor	*B*	SE	Wald	df	Sig.	Exp(*B*)
Preoperative CEA level	1.517	0.492	4.938	1	0.013	5.187
Degree of tumor differentiation	1.349	0.417	4.527	1	0.005	3.484
Lymph node metastasis	0.963	0.524	4.019	1	0.029	2.105
TNM stage	1.262	0.386	4.138	1	0.074	3.165

## Data Availability

The data used during the current study are available from the corresponding author.
